# A smartphone application for personalized facial aesthetic monitoring

**DOI:** 10.1111/srt.13824

**Published:** 2024-07-08

**Authors:** Wataru Hashimoto, Shohei Kaneda

**Affiliations:** ^1^ Mechanical Engineering Program Graduate School of Engineering, Kogakuin University Shinjuku‐ku Tokyo Japan

**Keywords:** automatic facial image capture, face alignment indicator system, facial skin, personalized facial aesthetic monitoring, smartphone, smartphone application, smartphone camera

## Abstract

**Background:**

Methods available at home for capturing facial images to track changes in skin quality and evaluate skincare treatments are limited. In this study, we developed a smartphone camera application (app) for personalized facial aesthetic monitoring.

**Materials and Methods:**

A face alignment indicators (FAIN) system utilizing facial landmark detection, an artificial intelligence technique, to estimate key facial parts, was implemented into the app to maintain a consistent facial appearance during image capture. The FAIN system is composed of a fixed target indicator and an alignment indicator that dynamically changes its shape according to the user's face position, size, and orientation. Users align their faces to match the alignment indicator with the fixed target indicator, and the image is automatically captured when alignment is achieved.

**Results:**

We investigated the app's effectiveness in ensuring a consistent facial appearance by analyzing both geometric and colorimetric data. Geometric information from captured faces and colorimetric data from stickers applied to the faces were utilized. The coefficients of variation (CVs) for the L*, a*, and b* values of the stickers were higher compared to those measured by a colorimeter, with CVs of 14.9 times, 8.14 times, and 4.41 times for L*, a*, and b*, respectively. To assess the feasibility of the app for facial aesthetic monitoring, we tracked changes in pseudo‐skin color on the cheek of a participant using skin‐colored stickers. As a result, we observed the smallest color difference ∆Eab of 1.901, which can be considered as the experimentally validated detection limit using images acquired by the app.

**Conclusion:**

While the current monitoring method is a relative quantification approach, it contributes to evidence‐based evaluations of skincare treatments.

## 1 INTRODUCTION

Facial skin quality undergoes a gradual decline with aging, yet it remains crucial for facial aesthetics due to its significant psychosocial impact on perceptions of age and health.^1^, ^2^ Daily skincare routines are essential for maintaining or enhancing facial skin quality, aiming to mitigate or reverse visible signs of aging.^3^ Monitoring these changes to evaluate the effectiveness of daily skincare regimens is essential for informed decision‐making regarding treatment continuation or discontinuation. While the VISIA Skin Analysis System provides sophisticated quantitative analysis and visual assessment of skin quality,^4^, ^5^, ^6^ portable three‐dimensional imaging systems like the LifeViz Mini^7^, ^8^ and Antera 3D^9^, ^10^ also offer quantitative insights. However, these professional‐grade systems, tailored for the beauty and cosmetic dermatology industries, are costly and impractical for daily home use by skincare consumers.

In contrast, the range of skincare products available for home use far surpasses the methods consumers have to assess visible skin quality. Leveraging smartphones for facial imaging presents a promising avenue, given their ubiquity and recent advancements in camera technology. Zhang et al. demonstrated the feasibility of quantitatively evaluating fine facial wrinkles using images captured by an iPhone 13 Pro Max.^11^ Nakashima et al. proposed a method for measuring skin transparency on the back of the hand using images from an iPhone 7.^12^ Li et al. developed a technique for measuring skin surface profiles to monitor skin lesions and mole development using images from an iPhone 13 equipped with an LED light dome.^13^ Hasegawa et al. introduced a method for capturing macro skin images using a smartphone with a ring light of LEDs, alongside an image conversion process to transform these into pseudo‐UV images using CycleGAN, a deep learning technique.^14^, ^15^

These endeavors mark significant progress in evaluating partial facial skin quality using smartphones. However, to achieve comprehensive facial aesthetic monitoring—a prerequisite for accurately gauging perceptions of age and health—a novel approach is imperative to standardize facial appearance conditions in images captured by smartphone cameras. Here, we introduce the face alignment indicators (FAIN) system, utilizing an artificial intelligence (AI) technique called Facial Landmark Detection (FLD),^16^, ^17^ to ensure consistent facial appearance during image capture. This system was integrated into an iOS camera application (app). In this study, we examined the consistency of facial appearance using geometric and colorimetric data from eight participantsʼ faces, acquired through successive images captured by the app. Additionally, we evaluated the feasibility of this app for personalized facial aesthetic monitoring suitable for home use by monitoring pseudo‐skin color changes on a participant's cheek using skin‐colored stickers.

## 2 MATERIALS AND METHODS

### 2.1 FAIN system and design of the app

The study utilized an iPhone 11 (Apple Inc., Cupertino, CA, USA) as the test smartphone. The camera app was developed as an iOS app using Apple's integrated development environment, Xcode (Apple Inc.), with Swift as the programming language. FLD, which estimates predefined landmarks (eyes, nose, mouth, eyebrows, and face outline) on facial images and provides geometric information,^16^ was employed to ensure consistent facial appearance conditions. Specifically, the VNDetectFaceLandmarksRequest class^17^ was utilized for FLD analysis within the Vision framework, Apple Inc.’s computer vision framework, to ensure uniform face appearance in each captured image. The FLD analysis yields XY coordinate information for 74 landmark points representing facial features when a human face is detected in the input real‐time video. It is worth noting that the accuracy of FLD analysis varies with facial orientations, with frontal faces yielding higher accuracy than sideways ones. In this study, four white points were utilized for the proposed FAIN system to achieve uniform facial appearance in images (Figure 1A). A triangle and straight line formed by these points (Figure 1B) serve as indicators for the FAIN system; one acts as a fixed target indicator, while the other serves as an alignment indicator that changes its shape to reflect variations in face size and orientation (Figure 1C).

**FIGURE 1:** The FAIN system, integrated into the app, ensures consistent facial appearance in captured images. (A) FLD analysis provides XY coordinate information for 74 facial landmark points. (B) The indicator consists of a triangle and a straight line connecting four white‐colored points from (A). (C) The FAIN system includes the target indicator (blue) and the alignment indicator (red) for face alignment. Photos of faces are used with permission by Generated Photos (https://generated.photos (accessed on 25 May 2024)).

Figure 2 depicts the workflow of facial image capture using the developed app. Initially, users verify whether the ambient light is 0lx using a digital illuminometer (78747; Shinwa Rules Co., Ltd., Japan). This step is crucial for standardizing illumination conditions during image captures, as demonstrated in our previous study, given its significance for relative quantitative color measurements of the captured image.^17^ Subsequently, the screen brightness is manually maximized using the brightness bar in the iPhone's Control Center before launching the app. Upon detecting a face, the FAIN system is activated, turning the screen white and displaying the indicators. This bright white screen also serves as an illumination source during image capture. Once face alignment is achieved, the front‐facing camera's shutter is automatically triggered to capture a facial image. The resolution and frame rate for the input real‐time video in the app are set at 1080p and 30 fps, respectively. Images captured using the app are saved in the RGB color space, specifically in the sRGB IEC61966‐2.1 profile, and stored in JPEG format with dimensions of 1080 × 1920 pixels.

**FIGURE 2:** Flowchart of the developed app. Tasks shaded in grey are performed by app users, while tasks in white, involving image capture for personalized facial aesthetic monitoring, are carried out by the app itself. During image capture, the display of alignment and target indicators is suspended.

### 2.2 Decision for completion of face alignment

Face alignment completion was determined using geometric information from both the target and alignment indicators. Here, the heights of the triangles for the target and alignment indicators are denoted as *h*_*T*1_ and *h*_*A*1_, respectively (Figure 1C). The bases of these triangles are represented by (*b*_*T*1_ + *b*_*T*2_) and (*b*_*A*1_ + *b*_*A*2_), respectively. Furthermore, the areas of the triangles are denoted as *A_T_* and *A_A_* for the target and alignment indicators, respectively. The centers of gravity for these indicators are referred to as *G_T_* and *G_A_*, respectively. Additionally, the lengths of the straight lines for both indicators are labeled as *h*_*T*2_ and *h*_*A*2_. Face alignment was deemed complete when the following five criteria were satisfied:

(1) $$\left(1\;-k\right)A_{T}\leq A_{A}\leq \left(1\;+\;k\right)A_{T}$$

(2) $$G_{\mathrm{Tx}}-k\left(b_{T1}+b_{T2}\right)\leq G_{\mathrm{Ax}}\leq G_{\mathrm{Tx}}+k\left(b_{T1}+b_{T2}\right)$$

(3) $$G_{\mathrm{Ty}}-k\;h_{T1}\leq G_{\mathrm{Ay}}\leq G_{\mathrm{Ty}}+k\;h_{T1}$$

(4) $$\left(1-k\right)b_{T1}/b_{T2}\leq b_{A1}/b_{A2}\leq \left(1\;+\;k\right)b_{T1}/b_{T2}$$

(5) $$\left(1-k\right)h_{T1}/h_{T2}\leq h_{A1}/h_{A2}\leq \left(1\;+\;k\right)h_{T1}/h_{T2}$$

where *G_Tx_* and *G_Ty_* represent the coordinates of the center of gravity of the target indicator triangle *G_T_*, while *G_Ax_* and *G_Ay_* denote the coordinates of the center of gravity of the alignment indicator triangle *G_A_*. The constant *k* takes values of 0.05 or 0.025 in this study. From a facial appearance standpoint, both the area *A_A_* and the center of gravity *G_A_* reflect the size and position of the face, defined by the relationship between the face and the smartphone camera.

### 2.3 Preparation of personalized target indicator and feasibility study of FAIN system

The feasibility of the FAIN system within the developed app was assessed using both a mannequin head as an in vitro face model (approximately 28.7 cm in height, Amazon Standard Item Number, ASIN: B08DY7BXPV) placed on a turntable (ASIN: B097C27663) purchased from Amazon Japan G.K., and eight participants. To generate individualized target indicators, facial images of the mannequin and participants were captured in advance using the default Camera app on the iPhone, referred to as the criterion image. Subsequently, geometric information of the four points (Figure 1A) was obtained using a laboratory‐developed FLD analysis app^17^ employing the same VNDetectFaceLandmarksRequest class. This information was then input into the developed app to create personalized target indicators. Facial images were captured under four conditions in this study. One condition relates to the smartphone's handling, either fixed to a camera tripod (“fixed”) or handheld (“hand”). The other condition pertains to face appearance criteria, either “tolerant” (with *k* set at 0.05) or “strict” (with *k* set at 0.025). For the fixed smartphone conditions, a tabletop camera tripod (Japanese Article Number: 4549892381157) purchased from Daiso Industries Co., Ltd. (Japan) was utilized.

### 2.4 Evaluation of app's usability and face appearance uniformity

To evaluate the app's usability, we examined the success rate of image capture within 120 s and the required capture time per image. Additionally, to assess facial appearance uniformity, we analyzed the geometric information of the face in images captured successively under the four conditions. The normalized area *A* was introduced to quantify the consistency of face size.

(6) $$A=A_{AA}/A_{T}$$

where *A_AA_* represents the area of the triangle of the indicator on the acquired images obtained by post‐FLD analysis using the laboratory‐made app. The distance *D* between *G_T_* and *G_AA_* was introduced to express the consistency of the face position as follows:

(7) $$D={\left\{{\left(G_{AAx}-G_{Tx}\right)}^{2}+{\left(G_{AAy}-G_{Ty}\right)}^{2}\right\}}^{1/2}$$

where *G_AAx_* and *G_AAy_* represent the center of gravity of the triangle of the indicator on the acquired images obtained by post‐FLD analysis. The normalized pitch *P* was introduced to express the consistency of the face pitch orientation:

(8) $$P=\left({h_{AA}}_{1}/{h_{AA}}_{2}\right)/\left({h_{T}}_{1}/{h_{T}}_{2}\right)$$

where *h*_*AA*1_ and *h*_*AA*2_ represent the height of the triangle and length of the straight line of the indicator on the acquired images, respectively. The normalized yaw *Y* was introduced to express the consistency of the face yaw orientation:

(9) $$Y=\left({b_{AA}}_{1}/{b_{AA}}_{2}\right)/\left({b_{T}}_{1}/{b_{T}}_{2}\right)$$

where *h*_*AA*1_ and *h*_*AA*2_ represent the lengths of the two distinct segments at the base of the indicator triangle in the acquired images. *b*_*AA*1_ and *b*_*AA*2_ intersect at right angles to the height of the triangle.

We also investigated variations in colorimetric information of the images as an indicator of facial appearance uniformity. Specifically, we utilized the L*, a*, and b* values in the CIELAB color space^18^ and the coefficients of variation (CV) of a cyan‐colored sticker affixed to the participant's faces. The cyan‐colored sticker (8‐mm in diameter; ASIN: B09C2Z3TVD) was procured from Amazon Japan G.K. The L*, a*, and b* values of the sticker (mean ± SEM) were measured using a portable colorimeter (WR‐10QC, Shenzhen Wave Optoelectronics Technology Co., Ltd., China) as a control, yielding values of 56.060 ± 0.082, −26.027 ± 0.133, and −25.031 ± 0.097, respectively (mean ± standard error of the mean (SEM), *n* = 25; involving 5 independent stickers measured 5 times each). A raster graphics editor (Photoshop 2024; Adobe Systems, San Jose, CA, USA) was employed to select and crop the sticker in the image as the ROI for color measurement. The selections were automated using the Magic Wand Tool in Photoshop. Color values over the ROI were measured, and their mean was calculated using the rgb2lab function in MATLAB (MathWorks, Natick, MA, USA).

### 2.5 Feasibility check of the app for personalized facial aesthetic monitoring

To assess the suitability of the app for personalized facial aesthetic monitoring, ultra‐thin, semi‐transparent, skin‐colored stickers (0.02‐mm thickness; ASIN: B0BVPS1TL7, SUHADA seal, Facelabo Co., Ltd., Japan) were obtained from Amazon Japan G.K. Two stickers, one in “natural beige” and another in ‘‘dark beige, referred to as patch1 and patch2, respectively, were utilized. These stickers were punched into circular shapes using an 8‐mm diameter biopsy punch (Kai Industries Co. Ltd., Japan) and then affixed to a predetermined area on the participant's cheek, demarcated by a blue‐colored plastic tape with a 15‐mm diameter aperture.

### 2.6 Data analysis

All statistical analyses were performed using a two‐sided Student's *t*‐test. In this study, *p* < 0.05 was considered significant.

## 3 RESULTS

### 3.1 In vitro and in vivo feasibility study of FAIN system

Initially, the feasibility of the FAIN system within the developed app was examined using a mannequin head (Figure 3 and Video S1). The alignment indicator's shape adjusted according to the face's size and orientation (Figure 3A), with the indicator changing from red to blue upon meeting face alignment criteria (Figure 3B–E). When the mannequin's face was undetected, the indicator and target marker displays were suspended (Video S1). The mannequin's facial images during various manual movements were captured using the app (Figure 4). Subsequently, the feasibility of the FAIN system for capturing facial images following human face alignment was assessed (Figure 5). During the face alignment process, the target and alignment indicators were displayed on a white screen within the app (Figure 5A and Video S2). Facial images were captured under four different conditions using the app (Figure 5B–E).

**FIGURE 3:** Confirmation of FAIN system operation using a mannequin head. (A) None of the criteria are met. (B) When the face pitch orientation criterion is met, the straight line in the indicator turns blue. (C) When both the face pitch and yaw orientation criteria are met, both the line and the outline of the triangle in the indicator turn blue. (D) When the face pitch orientation, as well as the size and position of the head criteria, are met, both the line and the interior of the triangle turn blue. (E) All criteria are met.

**FIGURE 4:** Facial images of the mannequin captured using the developed app. The images, obtained during (A) translational motion and (B) rotational motion of the mannequin head, were acquired under tolerance criteria (constant value, *k* = 0.05) for face alignment with the smartphone fixed on a camera tripod.

**FIGURE 5:** Facial images obtained using the app. (A) Sequential screenshots captured during face alignment using the app. The seconds indicated in the screenshots denote the time remaining before completion of face alignment and acquisition of the facial image (i.e., 0 s indicates the start of acquisition). (B–E) Images acquired under four different conditions. When the face alignment criteria were tolerant (constant value, *k* = 0.05), the smartphone was either (b) fixed to a camera tripod or (C) held by hand (i.e., variable smartphone position). When the criteria were strict (*k* = 0.025), the smartphone was either (D) fixed to a camera tripod or (E) held by hand.

### 3.2 Evaluation of app's usability, and face appearance uniformity

The impact of face alignment criteria and smartphone holding on the app's usability and facial appearance uniformity was assessed using images captured under four different conditions (Figure 6). The success rate for capturing within 120 s, serving as an indicator of app usability, indicated a significantly lower rate under the condition of strict face alignment criteria with a handheld smartphone (Hand/Strict) compared to other conditions (Figure 6A). The required capture time per image, used as a usability index, was notably shorter under the condition of tolerance criteria with the smartphone fixed to a camera tripod (Fixed/Tol.) compared to other conditions (Figure 6B). Distances between the center of gravity of the triangle in the target marker and the center of gravity of the triangles formed in the acquired images by FLD‐post analyses reflected the uniformity of captured face positions relative to those in the criterion image used to generate the target marker (Figure 6C). When closer to zero, these distances indicated closer alignment of faces in acquired images with those in the criterion image. Distances were significantly shorter when the smartphone was fixed (Fixed/Tol. and Fixed/Strict) compared to when held by hand with tolerance criteria (Hand/Tol.). Conversely, distances were independent of face alignment criteria when holding the smartphone by hand. The area of the triangle formed in captured faces by FLD‐post analyses was normalized to the area of the triangle in the target indicator to assess uniformity of face sizes relative to those in the criterion image (Figure 6D). When closer to 1, this normalized area indicated closer resemblance of face sizes in acquired images to those in the criterion image. Though a significant difference was noted between conditions where the smartphone was fixed and held by hand with tolerance criteria, no significant difference was observed between the condition where the smartphone was fixed with strict criteria, closest to 1, and the aforementioned conditions. Subsequently, color measurements summarized using L*, a*, and b* values of cyan‐colored stickers on faces in images revealed no significant differences among the four conditions (Figure 6G–I). Color uniformity within each participant's facial images was examined using coefficients of variation (CV) for L*, a*, and b* values, crucial for accurate facial aesthetic monitoring (Figure 6J–L). CV values closer to 0 indicate higher uniformity, with no significant differences observed among the four conditions. Table 1 compared color measurement variability under the four conditions with that of the control, representing values obtained from color measurements using the colorimeter. Smallest normalized CV values among L*, a*, and b* were observed under strict criteria with the smartphone fixed to a camera tripod (Fixed/Tol.). Conversely, largest normalized CV values were recorded under tolerance criteria with a handheld smartphone (Hand/Tol.).

**FIGURE 6:** Evaluation of app usability and facial appearance uniformity in images acquired under four different conditions. Points plotted in various colors represent results for each participant. When face alignment criteria were set as tolerant or strict, cases of a smartphone fixed with a camera tripod were denoted as (Fixed/Tol.) and (Fixed/Strict), and those of a smartphone held by hand as (Hand/Tol.) and (Hand/Strict), respectively. (N.S., not significant; *p < 0.05, **p < 0.01, *p < 0.001). (A) Success rate of capture within 120 s (*n* = 8, where *n* is the number of participants). (B) Time required for capture within 120 s. (C) Distance between the center of gravity of the triangle in the target indicator and triangles formed in the acquired images. (D) Area normalized by the triangle in the target indicator, reflecting the uniformity of face size in the images. (E) Normalized face pitch orientation. (F) Normalized face yaw orientation. (g–i) L*, a*, and b* values of cyan stickers on faces in the images (*n* = 40 (Fixed/Tol.), *n* = 39 (Hand/Tol.), *n* = 37 (Fixed/Strict) and *n* = 21 (Hand/Strict) for (G–I), where *n* corresponds to the number of images acquired under each condition). (J–L) Coefficient of variation of L*, a*, and b* values (*n* = 8 (Fixed/Tol., Hand/Tol., Fixed/Strict) and *n* = 4 (Hand/Strict) for (J–L)). Results for the four participants were omitted because the number of images acquired in (Hand/Strict) is two or fewer. Error bars indicate ± SEM.

**TABLE 1:** Variability of color measurements for cyan‐colored stickers on participants’ faces in the acquired images using the developed app. Control represents the coefficient of variation (CV) values obtained by measurements using the colorimeter (*n* = 5 (Control), *n* = 8 (Fixed/Tol., Hand/Tol., Fixed/Strict), and *n* = 4 (Hand/Strict), A two‐sided Student's *t*‐test was performed to compare each mean value under the four conditions with the control mean. An omission indicates no significant difference (*p < 0.05, **p < 0.01).

			95% CI		Normalized by control
Group	Mean	SEM	LB	UB	
CV of L* value					
Control	0.003042	0.001175	0.000740	0.005344	1.000
Fixed/Tol.	0.022951	0.009554	0.004224	0.041677	7.544
Hand/Tol.	0.045341	0.020247	0.005657	0.085026	14.904
Fixed/Strict	0.022218*	0.006420	0.009635	0.034802	7.303
Hand/Strict	0.016720*	0.005904	0.005148	0.028292	5.496
CV of a* value					
Control	−0.012874	0.009344	−0.031188	0.005441	1.000
Fixed/Tol.	−0.088586*	0.022340	−0.132373	−0.044800	6.881
Hand/Tol.	−0.104841*	0.024034	−0.151947	−0.057735	8.144
Fixed/Strict	−0.099970*	0.020345	−0.139845	−0.060094	7.765
Hand/Strict	−0.024880**	0.005558	−0.035774	−0.013986	1.933
CV of b* value					
Control	−0.010908	0.007010	−0.024649	0.002832	1.000
Fixed/Tol.	−0.024880	0.005558	−0.035774	−0.013986	2.281
Hand/Tol.	−0.048099	0.014099	−0.075732	−0.020466	4.409
Fixed/Strict	−0.031032	0.006102	−0.042991	−0.019073	2.845
Hand/Strict	−0.015320	0.005769	−0.026627	−0.004012	1.404

### 3.3 Feasibility check of the app for personalized facial aesthetic monitoring

Changes in skin color due to senile pigmentation, melasma, and sunburn are among the most evident indicators of alterations in skin quality.^18^ The app's potential for facial aesthetic monitoring was assessed by examining color measurements before and after affixing patches on the cheek to simulate pseudo‐skin color changes (Figure 7A–C). Significant differences in L* values were noted both between patch1 and natural skin and between patch1 and patch2 (Figure 7D). Moreover, significant disparities in the a* values were observed among natural skin, patch1, and patch2 (Figure 7E). In terms of b* values, significant differences were identified between patch2 and natural skin as well as between patch2 and patch1, while no significant difference was observed between natural skin and patch1 (Figure 7F). Table 2 details the color variations between natural skin, patch1, and patch2. It is important to note that ∆L*, ∆a*, and ∆b* represent absolute values, and if the confidence interval of a value includes 0, it is not considered in the calculation of ∆*Eab*. The most minimal color difference was observed between natural skin and patch2 (∆*Eab* = 1.901). The smallest ∆L* value was recorded between patch1 and patch2 (∆L* = 2.150), while the smallest ∆a* value was between natural skin and patch2 (∆a* = 1.236). Additionally, the smallest ∆b* value was noted between patch1 and patch2 (∆b* = 0.923).

**FIGURE 7:** Feasibility assessment of the app for personalized facial aesthetic monitoring. Representative facial images of (A) natural skin and simulated pseudo‐skin color changes using (B) patch1 and (C) patch2, acquired under tolerance criteria for face alignment with the smartphone held by hand. Arrows indicate the patches. (d–f) Color measurement results of L*, a*, and b* values. (N.S., not significant; ∗ *p* < 0.05, ∗∗ *p* < 0.01, ∗∗∗ *p* < 0.001; *n* = 5). Error bars indicate ± SEM.

**TABLE 2:** Color differences among natural skin, patches 1 and 2.

			95% CI	
	Mean	SEM	LB	UB
|ΔL*_(Native‐Patch1)_|	2.809	0.783	1.003	4.615
|Δa*_(Native‐Patch1)_|	2.986	0.257	2.393	3.580
|Δb*_(Native‐Patch1)_|	0.521^a^	0.297	−0.164	1.205
ΔEab*_(Native‐Patch1)_	4.100^b^	–	2.595	5.841
|ΔL*_(Native‐Patch2)_|	0.659^a^	0.525	−0.552	1.870
|Δa*_(Native‐Patch2)_|	1.236	0.312	0.516	1.956
|Δb*_(Native‐Patch2)_|	1.444	0.258	0.850	2.038
ΔEab*_(Native‐Patch2)_	1.901^b^	–	0.994	2.825
|ΔL*_(Patch1‐Patch2)_|	2.150	0.803	0.298	4.002
|Δa*_(Patch1‐Patch2)_|	1.750	0.353	0.936	2.565
|Δb*_(Patch1‐Patch2)_|	0.923	0.278	0.282	1.564
ΔEab*_(Patch1‐Patch2)_	2.922	–	1.022	5.004

^a^ Values with confidence interval includes 0.

^b^ Δ*Eab* values calculated without ΔL* or Δb* values whose confidence interval includes 0.

## 4 DISCUSSION

In this study, we developed a smartphone camera app designed to capture facial images for facial aesthetic monitoring by tracking changes in skin quality. To ensure precise monitoring, facial image captures were performed under standardized face appearance conditions using the FAIN system, which utilizes FLD and is integrated into the developed app. Additionally, these captures were conducted in complete darkness (0lx) to standardize illumination conditions.^17^ While conventional facial imaging systems^4^, ^5^, ^6^, ^7^, ^8^, ^9^, ^10^ boast higher precision than the proposed method, they are tailored for professional use, such as clinical applications by physicians or skincare product evaluation by developers. Conversely, our method is geared towards consumers utilizing skincare products at home, empowering them to conduct accurate self‐monitoring.

In the context of personalized facial aesthetic monitoring, the variability of color measurements in facial images captured by the app emerges as a critical index. As our method is not absolute quantification but relative quantification, and the distances between the camera and faces vary among participants, resulting L*, a*, and b* color measurements exhibit variability across individuals (Figure 6G–I). However, the examination of color measurement variability using CV values revealed no significant differences across the four conditions (Figure 6J–L). This implies that the observed significant differences in distance *D* and normalized area *A* (Figure 6C and D) do not impact the variability of color measurement outcomes. Consequently, tolerant criteria for face alignment deliver satisfactory quality for color measurements, akin to strict criteria. It is noteworthy that the normalized area *A*, pitch *P*, and yaw *Y* should ideally be included in alignment criteria (e.g., 0.95–1.05 when *k* equals 0.05). Instances where they fall outside the criterion range, as shown in Figure 6D–F, may be attributed to a time lag between the decision for face alignment completion and the app's automatic capture. To enhance color measurement precision, particularly for L*, the CVs for L*, a*, and b* values should be reduced (Table 2). According to our previous study on tooth color measurement, the L* value is most sensitive to changes in camera‐object distance.^17^ Tightening the criterion on the triangular area of the alignment indicator in the app would promote more consistent distance and improve color measurement accuracy.

The app's usability is as crucial as the variability in color measurement. Under tolerant conditions, the success rate for capturing images within 120 s showed no significant difference (Figure 6A). However, the time required per image capture was significantly reduced when the smartphone was fixed (Figure 6B). According to our preliminary study, the method of fixing the smartphone is not critical; simply leaning it against something effectively reduces the user's effort in face alignment, comparable to mounting it on a tabletop camera tripod (data not shown). This flexibility empowers app users to freely choose whether to fix the smartphone or hold it by hand, promoting personalized app usage without hesitation. While stricter criteria yield more consistent facial images, there's a trade‐off between success rate and capture time. Thanks to the automatic capture function implemented in the app, we were able to reduce the constant *k* to 0.05 in this study, compared to 0.3 in our previous manual capture study.^17^ This constant determines the consistency of the distance between the camera and faces, reflected in the normalized area, the most dominant factor affecting color measurement variability.

Our in vivo study, tracking pseudo‐skin color changes, demonstrated the feasibility of using the app for personalized facial aesthetic monitoring (Figure 7). Previously, P. Lagouvardos *et al.* reported that 50% perceptibility thresholds of facial skin color difference are as follows; ∆Eab* value of 1.497, ∆L* value of 0.119, ∆a* value 0.993, ∆b* value of 1.147, respectively^19^. The smallest color difference ∆*Eab* of 1.901, the minimum ∆L* value of 2.150, the minimum ∆a* value of 1.236, and the minimum ∆b* value of 0.923 respectively, observed in this study, can respectively be considered experimentally validated detection limits of using the app (Table 2). This suggests the app's potential for accurate monitoring of the ∆b* value, an index of pigmentation and tanning ability, especially for tracking changes in carotenoids, melanin synthesis, and oxidation after UV exposure, which are challenging to discern by the human eye.

Since the skin color in images captured by the app depends on the positional relationship between the camera and the subject, which varies among participants, our method is not absolute but relative, quantifying skin changes individually for each participant. Furthermore, because our method tolerates some inconsistencies deriving from the face alignment criteria, multiple facial images are required. In addition, our approach has several limitations. Firstly, it relies on the specific model of smartphone used, making comparisons between images obtained with different smartphone models unfeasible due to variations in camera and screen performance. Secondly, our method necessitates external software, namely Photoshop and MATLAB, for color measurements. Thirdly, our FAIN system is specialized for front‐facing faces, requiring different indicators for side‐facing ones. Additionally, our current FAIN system lacks criteria for mouth shape, leading to observed inconsistencies, which could affect color measurements. However, users can easily acquire facial images in selfie mode using only their smartphone, enabling them to assess skincare treatments independently, without advanced techniques or special equipment, and without assistance from others.

## 5 CONCLUSION

In this study, we developed a smartphone camera application for personalized facial aesthetic monitoring by tracking skin color changes. This app enables users to capture facial images in selfie mode with consistent face appearance, essential for assessing daily changes in facial skin quality autonomously. Despite the aforementioned limitations, this study lays the groundwork for evidence‐based evaluation of facial skincare treatments. Moreover, we believe that the potential applications of facial images acquired by the app extend beyond skincare assessment to include the accurate noninvasive monitoring of treatment responses for facial skin diseases^20^ and the rapid detection of signs of cognitive decline.^21^, ^22^

## CONFLICT OF INTEREST STATEMENT

S.K. has the following potential conflicts: CEO and equity holders at IQC Inc. W.H. declare no conflicts of interest.

## INSTITUTIONAL REVIEW BOARD STATEMENT AND INFORMED CONSENT STATEMENT

This study was conducted in accordance with the Declaration of Helsinki and approved by the Institutional Review Board of Kogakuin University (ref. no. 2020‐A‐4 and date 25 August 2020). Informed consent was obtained from all participants involved in the study.

## Supporting information

Video S1: Demonstration of FAIN system operation using a mannequin head.

Video S2: Facial alignment demonstration using the developed application.

## Data Availability

The data presented in this study are available upon request from the corresponding author.
